# Research on the Gas Emission Quantity Prediction Model of Improved Artificial Bee Colony Algorithm and Weighted Least Squares Support Vector Machine (IABC-WLSSVM)

This article has been retracted.

**DOI:** 10.1155/2022/4792988

**Published:** 2022-01-18

**Authors:** Lei Wang, Jinghang Li, Wenbo Zhang, Yu Li

**Affiliations:** School of Computer Science and Technology, Henan Polytechnic University, Jiaozuo, 454003 Henan, China

## Abstract

In order to further accurately predict gas emission of working face, this paper proposes a prediction model of gas emission of working face based on the combination of improved artificial bee colony algorithm and weighted least squares support vector machine (IABC-WLSSAVM). The research steps are as follows: Firstly, in order to obtain the sparse solution of LSSVM, a more reliable prediction model is realized by weighting the error value. Secondly, the chaotic sequence is introduced into the artificial bee colony algorithm to find a better initial honey source, which increases the diversity of the population, and combines the Levy flight to update the search step to avoid falling into the trap of local optimum. At the same time, the improved artificial bee colony algorithm is used to optimize the kernel width *σ* and regularization parameter *λ* of WLSSVM, which improves the prediction accuracy and convergence rate of WLSSVM. Finally, the quantitative analysis model of WLSSVM is reconstructed by using the optimized parameters, and the nine parameters of buried depth of coal seam, gas content of coal seam, coal thickness, interlayer lithology, production rate of working face, length of working face, inclination of coal seam, gas content of adjacent layer, and thickness of adjacent layer are used as the main influencing factors. After normalization, the nonlinear prediction model of gas emission is established. The simulation results based on the three indicators of determination coefficient, root mean square error, and average relative variance show that the IABC-WLSSVM prediction model proposed in this paper can not only overcome the local optimization to obtain the global optimal solution but also has faster convergence speed and higher prediction accuracy. This prediction model has obvious advantages compared with the other three improved prediction models in terms of fitting, accuracy, and generalization ability, which can provide a reliable theoretical basis for the prediction of gas emission in coal mining face under complex factors and propose a new idea for the application of artificial intelligence in the construction of intelligent mines. At the same time, the prediction model can also be applied to other fields.

## 1. Introduction

A gas accident is the main type of accident affecting coal mine safety production. In an effort to ensure the safety and health of workers and reduce the probability decrease, it is essential to make the coal mine risks known and controllable through certain technical means [1]. The prediction of gas emission is an important basis for modern mine construction, underground ventilation system design, and gas prevention. In large high gas mines, if the predicted gas emission is comparatively low or high, it will not only increase the operating cost of ventilation equipment, causing unnecessary waste, but also increase the safety hazard of underground workers. Therefore, the accurate prediction of gas emission has attracted much attention at home and abroad, and a variety of models have been established, including the mine statistics method, graphic source method, and gas geological mathematical model method [2–4]. The prediction results show that these methods are static prediction or point instead of surface prediction. The prediction results cannot reflect the actual situation of gas emission in production engineering of coal mining face with dynamic behavior, and the timeliness and reliability of prediction are poor. With the development of artificial intelligence technology, scholars in China and abroad have proposed many effective nonlinear prediction methods combined with machine learning algorithms for the improvement of gas emission prediction models [5], such as the CART regression algorithm [6], neural network [7], principal component regression analysis method [8], support vector machine (SVM) [9], and least squares support vector machine (LSSVM) [10]. These methods have achieved ideal results. A gas explosion is the most serious disaster in a coal mine, which is highly destructive and sudden, and often causes a large number of casualties and property losses. In the process of dealing with gas explosion accidents, if the treatment methods are improper and the key points are not grasped, multiple gas explosions may occur, resulting in the expansion of the accident.

However, the stability of the classical CART regression algorithm is relatively poor. Even if the data has a small change, the prediction results will be completely different. The neural network method is suitable for the scenario where the number of samples tends to be infinite, but it ignores the physical relationship between various influencing factors. When the number of samples is limited, the prediction effect is not ideal, and it is easy to fall into the local optimum. For the corresponding relationship between the influencing factors and related parameters established by the principal component regression analysis method, the fitting effect is not ideal due to the complex dynamic relationship between the influencing factors. SVM can effectively express the nonlinear relationship between data, which is more in line with the application of gas emission prediction. However, if the parameters are not properly selected, the accuracy of prediction will be relatively low. LSSVM is improved by Suykens et al. based on SVM. The model has the advantages of simple solution methods and fast calculation speed. Moreover, it has great advantages in dealing with nonlinear problems compared with support vector machines. Nevertheless, it lacks sparsity. At the same time, as with SVM, the prediction accuracy of LSSVM also depends on the selection of its parameters. If the selection is not appropriate, the accuracy will be relatively low. In recent years, some intelligent optimization algorithms have been successfully applied to model optimization, such as Qin and Fan [11] who built a support vector machine model based on the particle swarm optimization algorithm (PSO). Liu et al. [12] and Gu et al. [13] proposed the SVM parameter optimization method based on improved GA. However, these swarm intelligent optimization algorithms have many defects, such as too many parameter settings and complex optimization processes. The artificial bee colony (ABC) algorithm was first proposed by [14], which is a kind of biological intelligent optimization algorithm to simulate bee colony cooperation to find honey sources. It has many advantages, such as less parameter setting, simple calculation, high fitness, and strong robustness. In each iteration, both global and local searches are performed, and the global optimal solution can be quickly searched. Note that the generalization ability of the neural network algorithm means that it has good prediction ability and control ability for untrained samples. In particular, when there are some noisy samples, the network has good prediction ability.

This paper combines the improved artificial bee colony algorithm with the weighted least squares support vector machine (IABC-WLSSVM) to establish the prediction model of gas emission. The purpose is to improve the calculation speed of the prediction model and enrich the diversity of honey sources by introducing chaotic sequences so as to effectively avoid falling into the local optimal solution, thereby increasing the probability of obtaining the global optimal solution. Through the experimental simulation and quantitative analysis of nine key factors such as gas content of coal seam, production rate of working face, and thickness of adjacent layer, it is verified that the model can greatly improve the accuracy of actual gas emission prediction in the coal mine working face. The artificial bee colony algorithm is an optimization method proposed to imitate the behavior of bees. It is a specific application of the idea of cluster intelligence. Its main feature is that it does not need to understand the special information of the problem but only needs to compare the advantages and disadvantages of the problem. Through the local optimization behavior of each artificial bee individual, it finally makes the global optimal value emerge in the group and has a fast convergence speed.

## 2. Improvement and Performance Analysis of Algorithm

This section mainly introduces the optimization algorithm used in this paper and carefully analyzes the methods to improve the algorithm. At the end of this section, the improved artificial bee colony algorithm is optimized and compared in detail.

### 2.1. WLSSVM

The standard SVM model is very complex to solve the unknown parameters after duality transformation, especially when dealing with high-dimensional data. When a classification problem does not have linear separability, using hyperplane as the decision boundary will bring classification loss; that is, some support vectors are no longer located on the interval boundary, but enter the interior of the interval boundary, or fall into the wrong side of the decision boundary. The loss function can quantify the classified loss, and its form in a mathematical sense is 0-1 loss function. So, the model is difficult to promote. In view of this, Suykens et al. [15] proposed least squares support vector machine (LSSVM) and transformed the quadratic programming problem into solving equations by using the sum of error squares instead of the insensitive loss function of the support vector machine:

(1) $$\begin{array}{c} \min_{w,s,e}J\left(w,e\right)=\frac{1}{2}w^{T}w+\frac{1}{2}\lambda \overset{N}{\underset{i=1}{\sum }}e_{i}^{2}, \end{array}$$

(2) $$\begin{array}{c} y_{i}=w^{T}\psi \left(x_{i}\right)+s+e_{i}. \end{array}$$

In the formula, *w* is the weight variable, *λ* is the regularization parameter, *e*_*i*_ is the error value, *s* is the threshold, and *ψ*(·) is a nonlinear mapping in the kernel space. The optimization problem in the high-dimensional feature space involves complex operations and a large amount of calculation, which is usually converted into a dual problem. The Lagrange multiplier method is used to convert the original problem into the problem of finding the maximum value of the multiplier *α*_*i*_(*α*_*i*_ ≥ 0), and the following LSSVM decision function is constructed:

(3) $$\begin{array}{c} L\left(w,s,e,\alpha \right)=J\left(w,e\right)-\overset{N}{\underset{i=1}{\sum }}\alpha_{i}\left(w^{T}\psi \left(x_{i}\right)+s+e_{i}-y_{i}\right). \end{array}$$

According to the condition of extreme value, the partial derivative of the function to each variable is set to 0. And according to four conditions, we can list a system of linear equations about *α* and *s*:

(4) $$\begin{array}{c} \left[\begin{array}{cc} 0 & R^{T}\\ R & K+\lambda^{-1}I \end{array}\right]\left[\begin{array}{c} s\\ A \end{array}\right]=\left[\begin{array}{c} 0\\ Y \end{array}\right]. \end{array}$$

In the formula, *R* = [1, ⋯,1]^2^, *A* = [*a*_1_, *a*_2_, ⋯,*a*_*N*_]^*T*^, *Y* = [*y*_1_, *y*_2_, ⋯*y*_*N*_]^*T*^.

Although LSSVM effectively reduces the time complexity of SVM, the LSSVM model selects the least squares method to select the best, and assuming that the error value satisfies the Gaussian distribution, it will lead to biased estimation of parameters when the error value does not meet the assumption, and the model lacks robustness. Secondly, since the number of weight coefficients of the decision function is equal to the number of samples, the model lacks sparsity. To solve these two defects, Suykens et al. [16] proposed an optimization algorithm to improve the robustness and sparsity of LSSVM-WLSSVM. Using hard margin SVM in online inseparable problems will produce classification errors. Therefore, a new optimization problem can be constructed by introducing the loss function on the basis of maximizing margin. SVM uses the hinge loss function and follows the optimization problem form of hard boundary SVM.

#### 2.1.1. Improvement of Robustness

In order to prevent the influence of heteroscedasticity of error value on parameter estimation, the weight factor *v*_*i*_ is added on the basis of objective function [17] to improve the robustness of the model:

(5) $$\begin{array}{c} \min_{w^{*},s,e}J\left(w^{*},e\right)=\frac{1}{2}{\left(w^{*}\right)}^{T}w^{*}+\frac{1}{2}\;\lambda \overset{N}{\underset{i=1}{\sum }}v_{i}{\left(e_{i}^{*}\right)}^{2}, \end{array}$$

(6) $$\begin{array}{c} y_{i}={\left(w^{*}\right)}^{T}\psi \left(x_{i}\right)+s^{*}+e_{i}^{*}. \end{array}$$

In the formula, *w*^∗^ is the weight variable, *λ* is the regularization parameter, *e*_*i*_^∗^ is the error value, *s*^∗^ is the threshold, *ψ*(·) is a nonlinear mapping in the kernel space, and *v*_*i*_ is the weight factor, which is the function of LSSVM algorithm error sequence *e*_*i*_:

(7) $$\begin{array}{c} v_{i}=\left\{\begin{array}{cc} 1, & \left|e_{k}\sqrt{K}\right|\leq c_{1},\\ \frac{c_{2}-\left|e_{k}\sqrt{K}\right|}{c_{2}-c_{1}}, & c_{1}\leq \left|e_{k}\sqrt{K}\right|\leq c_{2},\\ 10^{-4}, & \text{otherwise}. \end{array}\right. \end{array}$$

In the formula, $\bar{K}=\text{IQR}/\left(2\times 0.6745\right)$, IQR is the difference between the third quartile and the first quartile after the error *e*_*i*_ sequence is arranged from small to large, and the values of *c*_1_ and *c*_2_ are 2.5 and 3, respectively.

Similarly, the objective function of WLSSVM can be obtained as follows:

(8) $$\begin{array}{c} L\left(w^{*},s^{*},e^{*},\alpha^{*}\right)=J\left(w^{*},e^{*}\right)-\overset{N}{\underset{i-1}{\sum }}\alpha_{i}^{*}\left({\left(w^{*}\right)}^{T}\psi \left(x_{i}\right)+s^{*}+e_{i}^{*}-y_{i}\right). \end{array}$$

And the new sequence of functions can be solved by

(9) $$\begin{array}{c} \left[\begin{array}{cc} 0 & R^{T}\\ R & K+V_{\lambda } \end{array}\right]\left[\begin{array}{c} s^{*}\\ A^{*} \end{array}\right]=\left[\begin{array}{c} 0\\ Y \end{array}\right]. \end{array}$$

In the formula, *V*_*λ*_ = diag{1/*λ*_*v*_1__, 1/*λ*_*v*_2__, ⋯, 1/*λ*_*v*_*m*__}, *A* = [*a*_1_^∗^, *a*_2_^∗^, ⋯,*a*_*N*_^∗^]^*T*^, *Y* = [*y*_1_^∗^, *y*_2_^∗^, ⋯,*y*_*N*_^∗^]^*T*^, *K* is the kernel function, and the radial basis function with a simple structure and good generalization performance is selected as the kernel function, which can be expressed as

(10) $$\begin{array}{c} K\left(x,x_{i}\right)=\exp\left(\frac{-\left\|x_{j}-x_{i}\right\|}{\sigma^{2}}\right). \end{array}$$

In the formula, *σ* denotes the kernel width. Some linear nonseparable problems may be nonlinear separable; that is, there is a hypersurface in the feature space to separate the positive class from the negative class. The nonlinear separable problem can be transformed into a linear separable problem by mapping the nonlinear separable problem from the original feature space to a higher dimensional Hilbert space.

#### 2.1.2. Improvement of Sparsity

Suykens proposes that parameter *α* can be optimized by selecting an optimization objective (such as accuracy); that is, the sparse model can be achieved by deleting sample points with small Lagrange multipliers, as formula (11) shows:

(11) $$\begin{array}{c} \alpha_{i}^{\text{new}}=\left\{\begin{array}{cc} \alpha_{i}^{*}, & \text{if }x_{i}\text{ is deleted},\text{the optimization goal is not enhanced},\\ 0, & \text{if }x_{i}\text{ is deleted},\text{the optimization goal is enhanced}. \end{array}\right. \end{array}$$

The optimal solution can be calculated by substituting the optimized *α* value back to formula (8).

After determining the kernel function, WLSSVM needs to further determine the parameters: kernel width *σ* and regularization parameter *λ*. And the IABC algorithm is used to optimize it.

### 2.2. Improvement of ABC Optimization Algorithm

Karaboga [14] proposed an optimization algorithm based on the bee colony intelligence-artificial bee colony algorithm. In this algorithm, the artificial bee colony algorithm is used to find the optimal honey source by simulating the different division of labor of the bee colony and exchanging the information of the honey source. Karaboga and Basturk [18], Karaboga and Basturk [19] through five common benchmark function test that the ABC algorithm has good optimization performance as the genetic algorithm and evolutionary algorithm.

However, although the ABC algorithm can easily obtain the optimal value, its population distribution is relatively single and the global optimization ability is limited, which is easy to fall into premature convergence. In order to make the algorithm achieve better search ability, this paper proposes a method to improve the artificial bee colony algorithm by combining chaotic sequences and adjusting step size based on Levy flight. At the same time, the improved algorithm is applied to optimize the WLSSVM model to achieve a better prediction performance.

#### 2.2.1. Introducing Chaotic Sequence

The population is initialized by using the randomness, regularity, and ergodicity of chaotic sequences, so that the initial individuals are uniformly distributed as far as possible, thus effectively avoiding local optimum. Through traversing and mutating the whole space of chaotic sequence, the diversity of the population is maintained and the precision is improved. At the same time, the chaotic interference is eliminated and the oscillation in the subsequent iterative process is avoided. The logistic map is a typical chaotic model in chaotic dynamics [20], and its expression is

(12) $$\begin{array}{c} x_{t+1}=\mu x_{t}\left(1-x_{t}\right). \end{array}$$

In the formula, the random number *x*_*t*_ ∈ (0, 1) and *μ* is the control parameter; when *μ* = 4, the system is in a completely chaotic state. In the iterative process, when the search number of the artificial bee colony algorithm is greater than the set maximum number and the better nectar source has not been obtained, it will fall into the local optimal solution.

In order to solve this problem, chaotic sequences are proposed to enhance the local search ability of the ABC algorithm. Randomly generate a new honey source as the initial condition of chaotic sequence *x*_0_ and normalize the initial value to (0, 1) before chaotic search, so when *t* = 0, a new source of honey is generated randomly, and the chaotic variable *S*_*j*_^*t*+1^ is iteratively calculated according to

(13) $$\begin{array}{c} S_{j}^{t}=\frac{x_{j}^{t}-x_{\min j}}{x_{\max j}-x_{\min j}}. \end{array}$$

In the formula, *t* = 0, 1, 2, ⋯, max, *x*_max*j*_ and *x*_min*j*_ are the upper and lower bounds of the *a*-dimension variable search. Formula (14) is brought into *s*_*j*_^*t*+1^ to generate a new source of honey. Then, calculate the fitness of the new honey source:

(14) $$\begin{array}{c} x_{j}^{t+1}=x_{j}^{\min}+s_{j}^{t+1}\left(x_{j}^{\max}-x_{j}^{\min}\right). \end{array}$$

Compare this value to the stagnation value. If the fitness value of the new honey source is greater than the current optimal solution, the optimal solution is replaced by the fitness value of the new honey source. Otherwise, let *t* = *t* + 1 be the chaotic variable *s*_*j*_^*t*+1^ generated iteratively again until the maximum number of searches.

#### 2.2.2. Search Behavior Based on Levy Flight

This paper extended the search range by introducing the Levy flight method [21]. When the search range falls into the local extreme, enlarge the search range and improve the search ability. Levy flight is a typical random step motion mode, which obeys Levy distribution, that is, the combination of short-range motion and a small amount of long-range motion.

The honey source based on Levy flight search behavior is updated to

(15) $$\begin{array}{c} {\text{v}}_{ij}=x_{ij}+\alpha \cdot \text{Levy}\left(u,v\right). \end{array}$$

In the formula, *x*_*ij*_ is the *j*-dimensional component of the honey source *i*, *α* is the step size factor, and Levy(*u*, *v*) is the random step size of Levy flight simulation using the Mantegna algorithm. The formula is

(16) $$\begin{array}{c} \text{Levy}\left(\lambda \right)=\frac{u}{{\left|v\right|}^{1/\beta }}. \end{array}$$

In the formula, *β* is a constant 1.5, (*u*, *v*) obeys normal distribution, *u* ~ *N*(0, *σ*_*u*_^2^),*v* ~ *N*(0, *σ*_*v*_^2^), where *σ*_*u*_ and *σ*_*v*_ are

(17) $$\begin{array}{c} \sigma_{u}=\left\{\frac{\Gamma \left(1+\beta \right)\sin{\left(\pi \beta /2\right)}^{1/\beta }}{\Gamma \left(1+\beta \right)\beta \cdot 2^{\left(1-\beta \right)/2}}\right\}, \end{array}$$

(18) $$\begin{array}{c} \sigma_{v}=1. \end{array}$$

The idea of Levy flight is used to enrich the diversity of the bee colony position and improve the search step length of the algorithm. So that the individual population has a certain chance to run out of the original small probability exploration area, expand the search range. Therefore, the intelligent optimization algorithm based on Levy flight is easier to jump out of the local optimal solution, which can effectively enhance the optimization ability of the algorithm.  Figure 1 is the design flow chart of using Levy flight update location in the artificial bee colony algorithm. The cuckoo search algorithm is a new metaheuristic search algorithm. The idea is mainly based on two strategies: cuckoo nest parasitism and Levy flight mechanism. Through random walk search, we can get an optimal nest to hatch our own eggs, which can achieve an efficient optimization mode. The main advantages of the algorithm are less parameters, simple operation, easy implementation, random search path optimization, and strong optimization ability.

### 2.3. Performance Test of the Improved Artificial Bee Colony Algorithm

The IEEE Conference on Evolutionary Computing (CEC2005) [17] held a real parameter function optimization competition and published 25 benchmark functions. Considering the running time, this paper uses 10 benchmark functions (F1-F12) to test the optimized performance of the ABC algorithm and IABC algorithm.  Table 1 gives the names, expressions, search spaces, and global optimal solutions of these 10 benchmark functions. According to the different characteristics of functions, these 10 functions can be divided into 2 categories: unimodal functions F1-F4 and multimodal functions F5-F10.

In order to ensure comparability and fairness, the initial values of the parameters of the colony algorithm are set in simulation experiment, as shown in Table 2. Because the IABC algorithm uses a more targeted population initialization method and a more scientific convergence method, the algorithm effectively avoids the local optimal conditions and achieves higher convergence speed.

In order to further compare the advantages and disadvantages of the IABC algorithm and the ABC algorithm, the 10 functions shown in Table 1 are used to test the optimization ability of the two algorithms in the 30-dimensional and 50-dimensional functions and record their optimal values, mean values, and standard deviation. The test results are shown in Tables 3 and 4.

It can be seen from the table that the IABC algorithm has higher comprehensive performance, and the standard deviation is lower than that of the standard ABC algorithm, which has higher calculation accuracy and stability. Among them, the reference function iteration diagrams of F1, F2, F5, F6, and F7 are shown in Figures 2–6.

From the matlab simulation results, it can be seen that the IABC algorithm improves the convergence accuracy of about 7%-14% than the ABC algorithm. Thus, it is verified that the artificial bee colony algorithm proposed in this paper can achieve better search ability by combining chaotic sequences and adjusting step size based on Levy flight. And it provides a strong guarantee for the optimization of the gas emission prediction model. There is another development feature of chaos theory, which has three principles: energy will always follow the path of minimum resistance; there is always a fundamental structure that is usually invisible, which determines the path of minimum resistance; and this always existing and usually invisible fundamental structure can not only be found but also be changed.

## 3. Construction of Model and Simulation Experiment

### 3.1. Construction of Gas Emission Prediction Model

The prediction model established in this paper consists of four main modules: preprocess module, test module, optimization module, and evaluation module. The specific steps are as follows:

**Step 1 (preprocess module).**

The normalization feature is a basic work of data mining. Different evaluation indicators often have different dimensions and dimensional units, which will affect the results of data analysis. In order to eliminate the dimensional impact between indicators, data standardization is needed to solve the comparability between data indicators. After data standardization, all indicators are in the same order of magnitude, which is suitable for comprehensive comparative evaluation. Because the feature vector in the sample space of gas emission has different physical meanings and dimensions, it is necessary to normalize the data before testing to improve the accuracy of prediction. The normalization interval of the data studied in this paper is [0.1, 0.9], and the normalization formula of the data is

(19) $$\begin{array}{c} Y=\frac{X-X_{\min}}{X_{\max}-X_{\min}}\times 0.8+0.1. \end{array}$$

In the formula, *X* is the original data of the current feature, *X*_min_ is the minimum value in the data, *X*_max_ is the maximum value in the data, and *Y* is the output value normalized. When the prediction process is completed, the data shall be denormalized, and the denormalized formula is as follows:

(20) $$\begin{array}{c} X=X_{\min}+\frac{\left(Y-0.1\right)\left(X_{\max}-X_{\min}\right)}{0.8}. \end{array}$$

**Step 2 (test module).**

Then, according to the principle described in Section 2.1, the WLSSVM model is constructed as the basic prediction model, and the optimized test results and analysis of input and output data are included later. Its structure is shown in Figure 7.

**Step 3 (optimization module).**

In this module, the penalty parameters *C*_1_, *C*_2_ and Gaussian kernel parameters *σ* of WLSSVM are optimized by the IABC algorithm, and the optimal parameter combination (*λ*, *σ*) is sought to maximize the regression accuracy of WLSSVM.

The establishment process of the IABC-WLSSVM model used in the optimization of gas emission prediction is as follows:

1. Select major influencing factors of gas emission quantity as training samples, normalize the original data by using the range processing method, and divide training samples and test samples
2. Initialize each parameter of the IABC algorithm according to the prediction model, and set the parameters such as the number of initial populations, the number of nectar sources, the maximum number of iterations, the number of cycle terminations, the number of hired bees, and investigation bees
3. Generate a number of initial populations through chaos sequence, select the best according to the distance function value, determine the corresponding population, and calculate the fitness value of each population to obtain the solution of the final initial nectar source
4. According to formula (15), the honey bees will find the new nectar source and find out the corresponding fitness. If the fitness of the nectar source is better than that of the original nectar source, the replacement operation will be carried out; otherwise, it will remain unchanged
5. Calculate the probability of all nectar sources being selected; then, the strategy of roulette was used to choose the nectar source and observe how the bees were collecting nectar and at the same time adjust the step size according to the Levy flight to search for new nectar sources nearby
6. Judge whether the cycle termination times are reached, and return to step (4) when the cycle termination times are less. If the fitness value of the nectar source does not change after the cycle termination times are reached, the investigation bee will give up the nectar source and produce a new nectar source
7. Output the nectar source solution corresponding to the maximum fitness value after the maximum number of iterations; otherwise, return to step (4) and continue searching
8. Put the optimal parameter combination solution (*λ*, *σ*) into the WLSSVM model, train with the test sample, obtain the solution, and put the parameters obtained into formula (14) to obtain the regression estimation function. The flow chart of the prediction model is shown in Figure 8

**Step 4 (evaluation module).**

In this paper, the coefficient of determination (*R*^2^), root mean square error (RMSE), and average relative variance (ARV) are selected as the criteria for evaluating gas emission prediction models.

*R* ^2^, also known as goodness of fit, determines the degree of correlation between the value estimated and the value measured. If the degree is close to 1, it can be indicated that the goodness of fit of data is good. If the degree is close to 0, it can be indicated that the goodness of fit of data is bad. The calculation formula is

(21) $$\begin{array}{c} R^{2}=1-\frac{\sum_{i=1}^{N}{\left(x_{i}^{`}-x_{i}\right)}^{2}}{\sum_{i=1}^{N}{\left(\overset{¯}{x_{i}}-x_{i}\right)}^{2}}. \end{array}$$

RMSE is the mean value of the square sum of error between predicted and measured values, which is generally used to evaluate the prediction accuracy of the model. The smaller the RMSE value, the higher the prediction accuracy of the model. The calculation formula is

(22) $$\begin{array}{c} \text{RMSE}=\sqrt{\frac{1}{N}\overset{N}{\underset{i=1}{\sum }}{\left(x_{i}-x_{i}^{`}\right)}^{2}}. \end{array}$$

ARV is used to judge the generalization ability of the model. The smaller the ARV value is, the stronger the generalization ability of the prediction model is. The specific calculation formula is

(23) $$\begin{array}{c} \text{ARV}=\frac{\sum_{i=1}^{N}{\left(x_{i}-x_{i}^{`}\right)}^{2}}{\sum_{i=1}^{N}{\left(x_{i}-\overset{¯}{x_{i}}\right)}^{2}}. \end{array}$$

In the formula, *N* is the number of samples, *x*_*i*_ is the original data value, *x*_*i*_^`^ is the sample predicted value, and $\overset{¯}{x_{i}}$ is the average value of the original data.

### 3.2. Simulation Experiments and Result Analysis

#### 3.2.1. Training of Sample Data

In this paper, 24 groups of measured data are randomly selected as the research objects according to the actual situation and main influencing factors in the field of Qianjiaying Mining Area of Kailuan Mining Group [22], wherein the first 15 groups of data are used as training data of the model, and the last 7 groups are used to test the accuracy of the prediction model of gas emission quantity. Cross-validation is not only a model selection method but also a model selection method that directly estimates the generalization error without any assumptions. Because there are no assumptions, it can be applied to various model selections, so it has universality of application. Because of its simplicity of operation, it is considered to be an effective model selection method.

There are many factors that affect gas emissions. In this paper, the following nine factors are selected for comprehensive consideration: buried depth of coal seam (*X*_1_/*m*), gas content of coal seam (*X*_2_/*m*^3^ · *t*^−1^), coal thickness (*X*_3_/*m*), interlayer lithology (*X*_4_), production rate of working face (*X*_5_), length of working face (*X*_6_/*m*), inclination of coal seam (*X*_7_/°), gas content of adjacent layer (*X*_8_/*m*^3^ · *t*^−1^) and thickness of adjacent layer (*X*_9_/*m*^3^ · min^−1^), and gas emission quantity (*Y*/*m*^3^ · min^−1^). The data of all influencing factors is shown in Table 5.

In order to normalize the sample data in Table 5, the parameter settings of the IABC-WLSSVM algorithm model are shown in Table 6. At the same time, the kernel width and the search range of regularized parameters are set as *σ*^2^ ∈ [0.01,5], *λ* ∈ [0.01,700], respectively. After the optimization of the IABC algorithm, the optimal parameters obtained by calculation are *σ*^2^ = 2.136, *λ* = 243.69.

#### 3.2.2. Prediction Experiment and Result Analysis of Gas Emission Quantity

Under the same training conditions, this paper applies the gas emission amount to the IABC-WLSSVM model, the genetic simulated annealing algorithm-regression support vector machine (GASA-SVR) [23], the support vector regression algorithm, the grey wolf optimization algorithm (GWO-SVR) [24], and the random forest algorithm model of improved artificial bee colony (IABC-RF) [25]. Under the same training frequency, the comparison results of the first 15 groups of training are shown in Figure 9.

From the comparison between the actual value of gas emission and the predicted value in Figure 9, it can be seen that the WLSSVM prediction model optimized by the IABC algorithm has a relatively higher fitting accuracy than the other three models. In order to better illustrate the performance effect of the prediction model, the last seven sets of data are selected for comparative analysis, and the performance of these prediction models is compared with *R*^2^, RMSE, and ARV.

It can be seen from Table 7 that in the 9 sets of measured data, the *R*^2^ value of the IABC-WLSSVM model is 8.44% higher than that of the GASA-SVR model, 8.07% higher than that of the GWO-SVR model, and 9.79% higher than that of the IABC-RF model. It shows that the predicted value of the IABC-WLSSVM model is closest to the real value compared with the other three models, and the overall goodness of fit is the highest.

From the perspective of RMSE, the RMSE value of the IABC-WLSSVM model is 54.31% lower than that of the GASA-SVR model, 54.57% lower than that of the GWO-SVR model, and 57.01% lower than that of the IABC-RF model. It shows that the prediction error of the IABC-WLSSVM model is significantly lower than that of other prediction models, which greatly improves the prediction accuracy of the model.

From the perspective of ARV, the ARV value of the IABC-WLSSVM model is reduced by 79.63% compared to the GASA-SVR model, 78.85% compared to the GWO-SVR model, and 81.67% compared to the IABC-RF model. It shows that the IABC-WLSSVM model has better generalization ability and its prediction model is more stable.

Figure 10 is a comparison diagram of the relative error rates of the four models. The relative error of each model can be calculated that the maximum error rate of GASA-SVR is 11.26%; the maximum error rate of GWO-SVR is 10.87%. Compared with the maximum error of the other three models, the prediction error of the IABC-WLSSVM model is the lowest, and the average error is only 3.29%. It indicates that the model has high fitting accuracy and can achieve ideal prediction effect.

Figure 11 is the convergence process diagram of the four model predictions. It can be seen from the convergence curve that the GWO-SVR model has basically completed the convergence after about 145 iterations, the IABC-RF model has basically completed the convergence after about 160 iterations, and the GASA-SVR model has basically completed the convergence after about 180 iterations. For the IABC-WLSSVM model, the convergence is basically completed after about 120 iterations, and the fitting error of the sample tends to be minimum. The curve shows that in the iterative process of IABC-WLSSVM, the nectar evolution quickly enters the convergence state and finds the optimal solution in the early stage, so that the individual fitness difference becomes larger in the later stage, and the premature phenomenon is avoided.

In order to more intuitively observe the difference between the predicted value and the real value of the model, according to the actual data of the 9 samples in Table 5, draw a histogram of the comparison between the true value and the predicted value. As shown in Figure 12, GASA-SVR models, GWO-SVR models, and IABC-RF models have large fluctuations between the real and predicted values, while the IABC-WLSSVM model has small fluctuations, indicating that the model can be as close to the real surge in real scenes as possible. The output value has high practical value.

## 4. Conclusion

In this paper, the improved artificial bee colony algorithm is organically combined with the weighted least squares support vector machine model to construct a new nonlinear gas emission prediction model based on IABC-WLSSVM. The model improves the sparsity of LSSVM by weighting the error value, thus optimizing the performance of the regression model. At the same time, the premature convergence problem of the ABC algorithm is improved by adding chaotic sequence and Levy fright method, which can effectively avoid the prediction model falling into local optimal solution, so as to obtain the global optimal solution more accurately. Then, the IABC algorithm is used to optimize the parameters in the WLSSVM model, and the optimized parameters are used to reconstruct the gas emission prediction model. Finally, the actual situation in the Qianjiaying mining area is applied as experimental data to this prediction model for simulation experiments. The data of nine main influencing factors, such as gas content of coal seam, production rate of working face, and thickness of adjacent layer, are input into the constructed model. The coefficient of determination (*R*^2^), root mean square error (RMSE), and average relative variance (ARV) were used as evaluation criteria for output and analyzed, respectively.

The experimental results show that the *R*^2^ value of the gas emission prediction model based on IABC-WLSSVM is 8.44%, 8.07%, and 9.79% higher than that of the GWO-SVR model, IABC-RF model, and GASA-SVR model, respectively, which indicates that the predicted value of this model is closest to the real value and the overall goodness of fit is the highest. The RMSE values were 54.31%, 54.57%, and 57.01% lower than those of the other three models, respectively. This indicates that the prediction error of this model is significantly lower than that of other prediction models, which greatly improves the prediction accuracy of the model. The ARV values of the three models are reduced by 79.63%, 78.85%, and 81.67%, respectively, indicating that this model has better generalization ability and is more stable in the prediction model, which effectively realizes the dynamic prediction of mine gas change trend.

The method is feasible and reliable and can be extended to other fields. However, this method also has some problems, such as the goodness of fit is not high enough. In the future study of gas emission prediction, we will analyze more gas emission data based on the measured data. At the same time, we will improve the existing model, such as using the adaptive ABC optimization algorithm to obtain more accurate prediction results.

## Figures and Tables

**Figure 1:** Flow chart of Levy flying bee colony algorithm.

**Figure 2:** Test results of F1 function.

**Figure 3:** Test results of F2 function.

**Figure 4:** Test results of F5 function.

**Figure 5:** Test results of F6 function.

**Figure 6:** Test results of F7 function.

**Figure 7:** WLSSVM prediction module.

**Figure 8:** Based on the improved IABC-WLSSVM algorithm flowchart.

**Figure 9:** Comparison of 15 groups of prediction results.

**Figure 10:** Relative error rate comparison chart.

**Figure 11:** Convergence process.

**Figure 12:** Line chart for prediction comparison of four algorithms.

**Table 1:** Benchmark function.

Benchmark function	Function	Remark	Optimal value	Benchmark function
F1	Sphere	$\text{F}1\left(x\right)=\overset{n}{\underset{i=1}{\sum }}x_{i}^{2}$	[−100, 100]^*D*^	0
F2	Quartic	$\text{F}2\left(x\right)=\overset{n}{\underset{i=1}{\sum }}ix_{i}^{4}+\text{random}\left[0,1\right)$	[−100, 100]^*D*^	0
F3	Bent cigar	$\text{F}3\left(x\right)=x_{1}^{2}+10^{6}\overset{n}{\underset{i=2}{\sum }}x_{i}^{2}$	[−1, 1]^*D*^	0
F4	Discus	$\text{F}4\left(x\right)=10^{6}x_{1}^{2}+\overset{D}{\underset{i=2}{\sum }}x_{i}^{2}$	[−10, 10]^*D*^	0
F5	Rastrigin	$\text{F}5\left(x\right)=\overset{n}{\underset{i=1}{\sum }}\left(x_{i}^{2}-10\cos\left(2\pi x_{i}\right)+10\right)$	[−5.12, 5.12]^*D*^	0
F6	Girewank	$\text{F}6\left(x\right)=\overset{n}{\underset{i=1}{\sum }}\frac{x_{i}^{2}}{4000}-5\overset{n}{\underset{i=1}{\prod }}\cos\left(\frac{x_{i}}{\sqrt{i}}\right)+1$	[−600, 600]^*D*^	0
F7	Rosenbrock	$\text{F}7\left(x\right)=\overset{n}{\underset{i=1}{\sum }}\left[100{\left(x_{i+1}-x_{i}^{2}\right)}^{2}+{\left(x_{i}-1\right)}^{2}\right]$	[−50, 50]^*D*^	0
F8	HappyCat	$\text{F}8\left(x\right)={\left|\overset{D}{\underset{i=1}{\sum }}x_{i}^{2}-D\right|}^{1/4}+\frac{\left(0.5\sum_{i=0}^{D}x_{i}^{2}+\sum_{i=0}^{D}x_{i}\right)}{D}+0.5$	[−30, 30]^*D*^	0
F9	Ackley	$\text{F}9\left(x\right)=-20\exp\left[-0.2\sqrt{\frac{\sum_{i=1}^{n}x_{i}^{2}}{n}}\right]-\exp\left[\frac{\sum_{i=1}^{n}\cos\left(2\pi x_{i}\right)}{n}\right]+23.1416$	[−32, 32]^*D*^	0
F10	HGBat	$\text{F}10\left(x\right)={\left|{\left(\overset{n}{\underset{i=1}{\sum }}x_{i}^{2}\right)}^{2}-{\left(\overset{n}{\underset{i=1}{\sum }}x_{i}\right)}^{2}\right|}^{1/2}+\frac{\left(0.5\sum_{i=1}^{n}x_{i}^{2}+\sum_{i=1}^{n}x_{i}\right)}{n}+0.5$	[−10, 10]^*D*^	0

**Table 2:** Artificial bee colony algorithm parameter setting.

Parameter	Value
Swarm size	50
Maximum number of iterations	300
Cycle termination times	100
Number of benchmark functions	5
Number of independent runs	30

**Table 3:** Performance comparison of ABC algorithm and IABC algorithm in 30-dimensional space.

Function	Algorithm	Optimal value	Mean value	Standard deviation
Sphere	ABC	0	4.17*e* − 16	3.28*e* − 16
	IABC	0	8.88*e* − 50	1.34*e* − 49

Quartic	ABC	1.443*e* − 02	8.603*e* − 02	3.233*e* − 03
	IABC	0	5.04*e* − 02	5.48*e* − 04

Bent cigar	ABC	3.67*e* + 02	4.86*e* + 01	1.77*e* + 01
	IABC	0	2.23*e* + 01	2.28*e* + 00

Discus	ABC	1.31*e* − 11	5.37*e* − 09	5.51*e* − 09
	IABC	1.06*e* − 21	8.47*e* − 08	1.42*e* − 18

Rastrigin	ABC	2.352*e* + 01	3.320*e* + 01	3.392*e* + 01
	IABC	0	5.08*e* − 02	2.04*e* − 01

Girewank	ABC	1.829*e* − 01	3.204*e* − 01	7.250*e* − 02
	IABC	0	2.66*e* − 17	1.33*e* − 16

Rosenbrock	ABC	6.618*e* + 01	1.374*e* + 02	1.056*e* + 01
	IABC	1.02*e* + 02	3.69*e* + 00	1.44*e* + 00

HappyCat	ABC	2.51*e* + 00	5.07*e* + 00	1.34*e* + 00
	IABC	0	2.61*e* − 09	4.89*e* − 17

Ackley	ABC	3.22*e* − 05	1.28*e* − 08	4.23*e* − 09
	IABC	3.73*e* − 13	1.36*e* − 09	1.68*e* − 15

HGBat	ABC	2.19*e* − 01	3.03*e* + 00	5.97*e* − 01
	IABC	0	2.53*e* − 18	6.92*e* − 07

**Table 4:** Performance comparison of ABC algorithm and IABC algorithm in 50-dimensional space.

Function	Algorithm	Optimal value	Mean value	Standard deviation
Sphere	ABC	1.728*e* − 01	1.341*e* + 00	2.713*e* − 01
	IABC	1.579*e* − 01	8.305*e* − 01	7.553*e* − 02

Quartic	ABC	9.127*e* − 01	2.124*e* + 00	1.344*e* − 01
	IABC	1.553*e* + 00	1.639*e* − 02	5.769*e* − 04

Bent cigar	ABC	8.28*e* − 12	4.01*e* − 09	1.77*e* − 11
	IABC	1.28*e* − 11	8.81*e* − 06	1.65*e* − 15

Discus	ABC	8.97*e* − 11	8.05*e* − 08	8.12*e* − 08
	IABC	1.11*e* − 22	7.11*e* − 18	2.804 − 09

Rastrigin	ABC	2.907*e* + 01	3.794*e* + 02	5.163*e* + 01
	IABC	1.647*e* − 02	4.681*e* + 01	8.803*e* + 00

Girewank	ABC	1.645*e* − 02	2.336*e* − 02	4.182*e* − 03
	IABC	9.332*e* − 03	2.047*e* + 00	1.515*e* − 03

Rosenbrock	ABC	1.978*e* + 02	1.978*e* + 02	2.465*e* + 02
	IABC	2.572*e* + 01	2.572*e* + 01	1.297*e* + 02

HappyCat	ABC	2.08*e* − 09	6.21*e* − 16	2.05*e* − 07
	IABC	1.16*e* − 17	4.11*e* − 18	5.63*e* − 09

Ackley	ABC	2.57*e* + 00	3.26*e* + 00	7.73*e* + 00
	IABC	1.16*e* − 16	1.24*e* − 13	3.95*e* − 15

HGBat	ABC	1.34*e* − 11	1.45*e* − 07	1.71*e* − 06
	IABC	5.85*e* − 22	4.74*e* − 18	1.26*e* − 07

**Table 5:** Original data of 9 main factors.

Number	*X*_1_	*X*_2_	*X*_3_	*X*_4_	*X*_5_	*X*_6_	*X*_7_	*X*_8_	*X*_9_	*Y*
1	408	1.92	2.0	5.03	0.96	155	10	2.02	1.50	3.34
2	411	2.15	2.0	4.87	0.95	140	8	2.10	1.21	2.97
3	420	2.14	1.8	4.75	0.95	175	11	2.64	1.62	3.56
4	432	2.58	2.3	4.91	0.95	145	10	2.40	1.48	3.62
5	456	2.40	2.2	4.63	0.94	160	15	2.55	1.75	4.17
6	531	3.35	2.9	1.82	0.93	165	9	1.88	1.42	4.78
7	516	3.22	2.8	4.78	0.93	180	13	2.21	1.72	4.60
8	527	2.80	2.5	4.51	0.94	180	17	2.81	1.81	4.92
9	563	3.68	3.0	4.53	0.94	175	11	3.11	1.46	5.56
10	550	3.61	2.9	4.83	0.92	155	12	2.12	1.60	5.23
11	634	4.80	6.5	4.62	0.79	165	9	3.02	1.74	7.68
12	590	4.21	5.9	4.77	0.79	170	8	3.40	1.50	7.24
13	640	4.67	6.3	4.60	0.80	175	11	2.56	1.75	7.95
14	604	4.03	6.2	4.70	0.81	180	9	3.15	1.80	7.80
15	634	4.80	6.5	4.55	0.73	175	12	2.98	1.92	8.51
16	509	3.24	2.5	4.65	0.93	160	14	2.79	1.72	4.36
17	580	3.87	3.9	4.72	0.92	170	11	3.02	1.39	5.82
18	635	4.53	6.2	4.61	0.72	160	9	2.94	1.73	7.56
19	629	4.62	6.4	4.63	0.81	170	13	3.35	1.61	8.04
20	544	3.16	2.7	4.90	0.93	165	17	2.81	1.79	4.93
21	450	2.43	2.7	4.58	0.93	165	11	2.35	1.85	5.06
22	640	4.67	6.3	4.60	0.80	175	11	2.56	1.75	7.95
23	415	2.46	2.3	4.68	0.96	158	11	2.42	1.23	4.07
24	556	3.37	2.7	4.49	0.93	165	13	1.88	1.42	4.78

**Table 6:** Parameter setting of IABC-WLSSVM model.

Parameter	Value
Initial population	80
Swarm size	60
Pick bees	30
Watch bees	30
Maximum number of iterations	100
Maximum number of chaotic iterations	200
Cycle termination times	50

**Table 7:** Comparison of prediction performance of four algorithms.

Model	Number	Truth value	Predictive value	Relative error (%)	*R* ^2^	RMSE	ARV
GASA-SVR	16	4.36	4.74	8.72	0.9036	0.4642	0.0054
	17	5.82	5.32	8.59			
	18	7.56	7.03	7.01			
	19	8.04	7.65	4.85			
	20	4.93	4.51	8.52			
	21	5.06	5.63	11.26			
	22	7.95	7.34	7.67			
	23	4.07	4.39	7.86			
	24	4.78	5.15	7.74			

GWO-SVR	16	4.36	4.81	10.32	0.9067	0.4568	0.0052
	17	5.82	5.46	6.19			
	18	7.56	7.93	4.89			
	19	8.04	7.56	5.97			
	20	4.93	4.47	9.33			
	21	5.06	5.61	10.87			
	22	7.95	7.36	7.42			
	23	4.07	4.42	8.60			
	24	4.78	5.22	9.21			

IABC-RF	16	4.36	4.76	9.17	0.8925	0.4934	0.0060
	17	5.82	5.47	6.01			
	18	7.56	8.04	6.35			
	19	8.04	7.59	5.60			
	20	4.93	4.52	8.32			
	21	5.06	4.72	6.72			
	22	7.95	7.08	10.94			
	23	4.07	4.48	10.07			
	24	4.78	5.27	10.25			

IABC-WLSSVM	16	4.36	4.46	2.52	0.9799	0.2121	0.0011
	17	5.82	5.54	4.98			
	18	7.56	7.72	2.38			
	19	8.04	7.82	2.86			
	20	4.93	5.13	3.86			
	21	5.06	4.87	3.36			
	22	7.95	7.57	4.91			
	23	4.07	4.17	2.46			
	24	4.78	4.89	2.30			

## Data Availability

The data underlying the results presented in the study are available within the manuscript.
